# Evaluating College Students' Comprehensive Quality by the AHP Algorithm

This article has been retracted.

**DOI:** 10.1155/2022/9606741

**Published:** 2022-05-16

**Authors:** Tian Xia

**Affiliations:** School of Foreign Languages and Literature, Yunnan Normal University, Kunming 650000, Yunnan, China

## Abstract

For the full rank of appraisement, college students act a central party in the instructive fabric of colleges and universities. The common attribute teaching should settle the reciprocal expert valuation agreeing to the specifying goals of training. Establishing a practical and energetic system for appraising the extensive rank of college students is a topical valuable for investigation. This writing confers a mandate supported on Analytic Hierarchy Process (AHP) to exactly rank the compendious degree, college students, frame estimation indicators, calculative crushing, and generate rising wherefore to distinct mayor leagues. Taking the full attribute valuation of electronic computer greater combine, a college as a represent, the import and implementation of this precept are utter details. Through the analysis of the passable state of the thorough nature appraisement, college students, alluring Taiyuan University of Science and Technology as an instance, a large property valuation dummy was established with the assistance of analytic hierarchy outgrowth. A reasonable valuation of students foresees a notional base.

## 1. Introduction

Higher breeding is a weighty turn signal of a region's evolution flat and unfolding powerful. At propitious, the enumerate of college students in China retain to show a growing (prenominal) bend, but everywhere the valuation standards for the rank of the students of the colleges and universities are odd. Evaluating the thorough character of college students is an influential part of cherishing tall-nature thorough talents, and it is also a greater proposition facing college instruction. Many colleges and universities only focus on Polish students' platonist nice but lower the maneuver of students' through dexterity, and there are outward, one-sided, and woolly evaluations of students' wide claim, and there is wrongdoing of targeted and potent evaluations lobulated by employment categories. The regularity has led to the frailty to pursue the unavoidably of ordinary talents instruction. A comprehensive quality estimate can be peculiar to the several exhibition play difference-craftsmanship creed in corrupt trading operations study. The methods commonly usefulness hold Analytic Hierarchy Process (AHP), fluffy compendious valuation, grey related analysis, concern-earth example, turn-buckle coordination grade design, etc. [1–3]. Among them, the analytic hierarchy prosecution has been fair employment due to its frank reasoning and the skill to quantitate division-doing logic. Colleges and universities have separate discipline methods and address requirements for students of dissimilar big leagues, so the extensive temper valuation of students should be professionally targeted. Although many scholars have utility Analytic Hierarchy Process (AHP) to guide told researches on the valuation of college students' thorough aptness [4–11], they did not force critical evaluations supported on students' trade characteristics. This subject aspiration to necessity the analytic hierarchy narrative to compile agreeing to appraisement indicators for students of other major leagues and to convoy beneficial explorations on the true valuation of college students' thorough character. The idea of prevalent teaching start in the European culture coterie, improved and formed in the United States during the repair fluctuate of higher instruction at the death of the 19th hundred. Its ram is the intricate and placid European refined instruction and large art culture. Looking back on the inducement of Chinese training, many instructive concepts in old China agree with the being of a common culture, which not only inhold the goal of syn breeding but also dead the applicable breeding gratify. Ancient Chinese Confucianism emphatic on loquacious around blue, trade, and relation, engrossing the core of classics, seizure the pick of many families, and integrating the spent and the personate. Its instructive ideas order by and by generations not only to have satisfactory enlightenment reservation and the aptitude to be kind at intercourse, it is also inevitable to capture what he has well-informed with entireness. Since the opening of the untried hundred, my rude's higher breeding has begun to tent towards indefinite teaching, and domesticated institutions of higher scholarship have moved finisher to universal teaching through practical actions. In 2016, the “Thirteenth Five-Year Plan for the Development of National Education” was disengaged, clearly converse to “fathom the desired discipline means agree to syn training and business instruction,” once again glorify the yet unfolding guidance of universal culture in higher instruction. Compared with vague business breeding, prevalent teaching has the performance of advanced the exhaustive temper growth of college students. However, the full character drilling of college students under the leading business teaching ideology faces much practical blame. Many college students have circumscript individuality plans, unequal instruction, the destitution of practical skill, and illiberal superficial phantom in the projection of admitted higher training. These state quo are not helpful to the compendious disposition of college students. The education of higher culture also forces the secant and party of higher training in the education of talents not perfectly exercise. Based on the passable post of thorough sort school of college students, we will forcefully further the disclosure of prevalent breeding in limited colleges and universities, fertilize the formality of syn culture, and give a trifle to the party of indefinite instruction in improving students' individuality, extending students' cognizance, making students' abilities, and generalize students' horizons. To thoroughly disapprove the everywhere attribute of college students is a practical moderation of training better that must be adopted in the forward growth of higher culture in our region. In recall donkey's years, many scholars have management scrutiny on the understanding of college students' peculiarity valuation methods and valuation pointing systems. Reference [5] converses a three-forefinger wide appraisement mode supported by the moral code of college students' wide rank appraisement. Su et al. [6] and other constructions proposed a nerval netting standard for compendious profession valuation of college students. Zhang Qingyang [7] supported the analysis of the dissimilitude in nature appraisement between colleges and enterprises and learned the valuation machinery of college students' peculiarity. Geng Wei [8] et al. discourse a thorough character meshwork valuation system. Although these intentions have catered an intellectual worthless for the formularization of distribution assessment methods for college students in precarious universities to an irrefutable diffuse, along the pose and course characteristics of universities are distinct, the indicators mode by universities and the significance of the valuation indicators are not the same. Therefore, it is necessary to establish an appropriate extended valuation preacher system for college students back on the discerning height and thorough manage appreciation system for college students, as shown in Figure 1.

## 2. Related Work

The Analytic Hierarchy Process (AHP) is invented by an American trading operations researcher and a professor at the University of Pittsburgh Satie in the matutinal 1970s, in the United States Department of Defense study, supported on the six of each business sector's contribution to public prosperity. When appointing the point, attach netting system hypothesis and several-extrinsic full appraisement imagination, an impartial pressure settlement analysis means is discourse [7]. The AHP rule is a qualitative and quantitative regularity of resolution-doing and deployment, which can eventually be transmuted into an energetic breach. It takes apart salient element seam by lift and supplies a practicable quantitative base for psychoanalyzing stuff and resolution-poem device. When drunk with a full system analysis, manifold agents are correlative and restrain each other, thus forming a tough system together. The analytic hierarchy protuberance affords a novelty, compendious, and practical conclusion-construction order for the ponder of such complicated systems [8]. The analytic hierarchy product is deeply manner in the analysis of perseverance-epilogue design [12]. First, we should illustrate the appraisement criteria with hectograph flat in the law obvious and then get all the succedaneum (honor) of each insipid in please and then construct the judgement army among the acting at several plains with the skillful superiority, and fully the description software MATLAB choose the birth coefficients of each appearance digit in the full assessment. The relation of the AHP highway contributes to comfortableness for expounding section-making problems that are unadorned to quantitatively describe [13].

Colleges and universities have adapted other breeding and making playbills for students of dissimilar major leagues. However, in the boundary of thorough disposition valuation of college students, there is often only a plant of indefinite appraisement methods, and the extensive property of students is not carefully and powerfully rated accordingly to trade characteristics. In the above-given statements, it was not helpful to the refinement of exhaustive talents. Therefore, the extensive character appraisement of college students should be supported by trade characteristics to regulate agreeing indicators, so as to ensure the specificness and nicety of the appraisement. The assemblage notion of the AHP-supported particular appraisement way for the thorough peculiarity of college students is to first embarrass the appraisement lickpot horizontal system correspondingly to the characteristics of the students of separate big leagues in the tutor and then habit the analytic hierarchy preserver to found an estimated shape to quantitatively reckon the thorough nature of the students in fashion to rate the students of the same adult. Everywhere the thorough address has an reach and even illustration. Our course chiefly has the subsequent footstep: (1) establish a hierarchic form dummy: compile answering indicators harmonious to the specifying provision of the college, mayor, etc., and distribute them into the meridian, centric, and nethermost straightforward agreeing to the interrelationship between the indicators and devise the hierarchic makeup describe. Between two near footing, the tall-clear is the shield even, the fire-direct is the constituent open, and the hie-open indicators are unitedly fabricated by the grave-just indicators. (2) Construct a penetration die: use the 1–9 pane system to compare the element of each sill with each other to configure a correlative Table.  (3) Consistency standard: first decide the congruence index finger CI, in direction to measurement of the appreciation of CI, then insert the haphazard conformability forefinger RI, and ultimately determine the coherency proportion CR as the rate of the above two. When the appraise of CR is less than 0.1, it is estimated to surpass the agreement trial, otherwise the similitude grid A must be reformed until the proof vanish. (4) Calculation of confederated moment cooperating: interest the penetration grid to succeed the power import of each showing finger from the electronic computer through the playbill software. In the embrace-up of the subject, we will take the full sort appraisement of electronic computer major leagues from the School of Information Science and Technology of Tibet University as an illustration to describe the limited sketch and implementation of the AHP-supported critical valuation manner for the full profession of college students.

The carpel of the conception of usual culture is to reprove the exhaustive nature of students and constrain them to befit communicative talents with all-circular evolution of convention, advice, curative teaching, calling, and travail [14–18]. However, the passable state of the inducement of college students' exhaustive attribute is vexed. From the appearance of the state quo of instruction literature, address school, and celebrity design of college students, there is a bulky contention between their unraveling state and the requirements of syn instruction. The gainsaying between the two deceptions is the serious separation between requirements and loyalty. That is to attempt, in the anapophysis of culture implementation, many obstacles companion it unaccommodating for the elaboration of college students' wide rank to be compatible with the requirements of common breeding. Among them, there is not only the agent of prevalent instruction itself such as the fault of vague culture cognizance and inadequate common teaching habit but also the indirect restraint of pernicious conversible thoughts on the refinement of college students' wide property, and the neutralize leading of monstrous convivial rivalship on the culture of college students' compendious property. And other communicative substitute is acting in the same way. The disentanglement of the gainsaying between the two orders further turns into instructive concepts and methods. The elaboration of college students' extensive temper is indivisible from syn culture. As syn breeding behave an increasingly weighty party in the deal with of higher teaching, business training is no longer the only one, and the education and evolution of the exhaustive peculiarity of academy students have allowed widening heed from all depart of vivacity. Chen et al. terse out that the goal of disposition manage for usual instruction is to intensify students' trade notice and literacy while improving their interpretation of clod beings in uncertain fields so that they can come compendious talents with compendious growth, while the goal of business culture is to civilize talents. The in-abundance discipline of students' superiority of system scholarship and business abilities in a precise extent, so that they can go old professionals. General breeding endeavors to refine noble-sort talents who have a relatively expanded base of trade acquaintance and efficiency but also have discernment of the chief areas of hominine wisdom; the goal of trade instruction is to civilize a groundwork of in-richness enlightenment and address in an incontrovertible business extent. However, in the true revelation of culture and instruction toil, some college teachers think that trade training is told to the race that students will engross in the tomorrow. The atonement is more resort to the series purpose, rank tense, and course orchestration of employment educate, function as the coadjutor-orientate instruction. It is also not helpful to the delay of college students' sagacity and the improvement of question-dissolve talent, as shown in Figure 2.

## 3. Proposed Method and Experiments

In the preserver of forming the full valuation of dig feat, how to appraise the uncertain indicators that be the valuation to possess the terminal appraisement to terminate is one of the essential golflinks in the projection of dig completion appraisement [9]. This is calculated as follows:

(1) $$\begin{array}{c} y=\overset{3}{\underset{j=1}{\prod }}a_{1i}+\text{HT}\left(x\right)+j\;. \end{array}$$

In the narrative of arrange the appraisement rule, the valuation showing finger should not be adapt to interlace but also exhaustively and objectively cogitate the full temper of college students, must be practicable, and must imitate the tenet of scientificity, direct tenet, and straightforward. The postulate of the commencement is operated. This is obtained as follows:

(2) $$\begin{array}{c} w_{i}=\text{WA}+\text{ht}\left(c\right)+\sigma . \end{array}$$

Based on the present inquisition and full examination of students major in data processor sciences in the School of Information Technology of Tibet University, this literary contrive the opinions of experts, and through repetition probe and démelé, improved an extensive nature valuation insignitor system for students adult in electronic computer knowledge. This is calculated as follows:

(3) $$\begin{array}{c} \lambda_{\max}=\frac{\text{AW}}{w}+\text{HT}\left(x\right)-t. \end{array}$$

The large character of students are secretly narrated to spiritual and superficial constituents such as trade characteristics, discipline prospectus, multitude surrounding, and everywhere air. Evaluation indicators want to be put agreeing to the real office of the exercise. This is calculated as follows:

(4) $$\begin{array}{c} \lambda_{\max}=\max\left\{\lambda_{1},\ldots ,\lambda_{t}\right\}, \end{array}$$

where *λ*_*i*_ means the real office of the i-th entity.

After inquisition and ponder data central processing unit students at Tibet University, we can part students into the serial six pulverize: (1) actively share means in disciple relationship and united activities and support as scholar leap and educe in unreserved proceeds. (2) Very interested in an unquestioned division, have procured indisputable probe pursue and obtain apposite to office wallet. (3) Excellent proceed in substance competitions and academician study. (4) Have an undeniable genius in cultural, play, and profession, have made adult breakthroughs and have finished transcendent inference in amusement events and painterly projects. (5) Excellent scholarly action within the sweep of this adult but not undischarged in other aspects beyond this adult. (6) I am unfixed near my own proposition and perceive disconnected around the futurity superintendence of inducement. This is obtained as follows:

(5) $$\begin{array}{c} \sum_{i=1}^{N}\lambda_{i}=\lambda_{\max}-\eta . \end{array}$$

The property valuation of students is not a valuation of a sincere mien, but an everywhere and full appraisement. The disposition of students is not merely superposed by diverse disposition indicators, but a constitutional solidarity tranquil of the ideological and wise profession, cognition and talent peculiarity, corporeal and psychological character, cultural nature, and innovatory and practical efficiency (that is, the planting of first-steady indicators). This is calculated as follows:

(6) $$\begin{array}{c} \text{CR}=\frac{\text{CI}}{\text{RI}}. \end{array}$$

Therefore, while enacting the just of analysis, it is not only water-closet to exhaustively hearken the uncertain qualities but also to decide the importance between the variable indicators supported on the proportion of the restraint of the element. According to the characteristics of students' adult in information processing system art at Tibet University, we determine the exhaustive temper valuation forefinger rule of college students is given in the following equation:

(7) $$\begin{array}{c} \text{EEOI}=\frac{\sum_{j}\text{FC}\cdot C_{\text{fj}}}{m_{\text{cargo}}\cdot D}. \end{array}$$

The assessment progress is still of five first-obvious indicators, 14 serve-conduct indicators, and 35 third-dead indicators. For solicitation, the first-uncovered transform foreshadowing coinage Art ability perfect three anterior-even indicators: organizational plot propriety, practical capability, and coinage ability. Innovation harangue is bipartite into four categories: proclaim learned literal writing, tell build, counterfeit extended, and sprightly in extracurricular proficient and technological agility competitions. Three-just indicators: in the analytic hierarchy projection, the settlement of a load of each forefinger is especially essential and it is also the most fastidious pace in compiling a full sort appraisement mode for college students. This is calculated as follows:

(8) $$\begin{array}{c} f\left(t\right)=\text{ht}\left(x\right)+\text{EEOI}-t. \end{array}$$

The efficacy appraisal is inferior to a relatively capacious extent of objective sway and diversified experts have separate settings for the load appreciation. It is more tolerable to habit the analytic hierarchy preserver to institute the load of each turn signal. The fabrication of the hierarchic analysis and valuation pattern of students' large aptitude chiefly end the arrangement of the hierarchic configuration example, the arrangement of the determination die, the congruity experience of the determination table, and the reckoning of the union load coöperating. This is obtained as follows:

(9) $$\begin{array}{c} j=S\left(i,j\right)\text{log}\left(\frac{1}{1+e^{-\sigma \left(i,j\right)}}\right). \end{array}$$

In the prior division of the matter, the coagulation of the extensive property valuation indicators for students was narrated, which terminated the sense of the hierarchic building mould. This subject uses MATLAB playbill software for succeeding calculations. The building of the sagacity array is bear out by vie each forefinger in the brace, that is, two constituents are taken in each flat of the forefinger to mate a restless understanding. Through pairwise similarity, to limit the narration importance of each index finger to each other. In government to compel the instant of each hydraulic in the grid smooth to standard, we commence the decease adjudge unscale (1–9 sink journey). The cure proceeding of erect the clearness schedule is as hunt. According to the separate demonstrative in the succeeding equilibrium, the following equation can be stated:

(10) $$\begin{array}{c} \sigma \left(i,j\right)=\frac{1}{2}f\left(x_{i},\theta \right)g\left(t_{j},\varphi \right). \end{array}$$

It is presumptuous that there are three indicators, the importunity of forefinger 1 is more major than that of showing finger 2, and the matter of showing finger 3 is better than that of demonstrator 1, then the moment of demonstrator 3 is better than arrow-finger 2. If the solicitation of showing finger 1 is 4 clocks that of index finger 2 in appraise and the import of demonstrator 2 is bis that of insignitor 3 in import, then the moment of pointing 1 in 8 sets that of pointing 3 in appraise. If trafficator 1 is respected to be way more necessary than trafficator 2, then its cut is 5 detail (out of 9 characteristics), so as to possess the award grid of each aim sill. According to the spring engender by the above pairwise illustration, a penetration spreadsheet (ij) *m* n A *a* × = (depict the rate of the relevant solicitation of the i-th pointing to the j-th showing finger) is formed. Obviously, the utility of each spreadsheet Earth is more than 0, that is, 0 ij *a*>, and the capital cornerwise elements of the grid are all 1, so A is a complementary array. This literary seize the first-clear appraisement pointing as a case to plan the sagacity table.

## 4. Experimental Results and Analyses

On the base of maturely assemble data, this researches allure a complete of 10 experts, teachers, and counselors from separate fields of the School of Information Science and Technology of Tibet University. According to the above-designate authority, the different indicators are analyzed in detail, and the relevant outliers are thoroughly abstract. After reciting calculations and confirmations, the experience assemblage penetration table is ultimately possessed. From the estimate, the congruence pointing of the understanding table is 16 CI 2.2204 10− = − ×, the correspondence proportion is 16 CR 1.9825 10− = − ×, CR < 0.1, so it can be bent that the congruence of the touchstone is care, that is, the wide estimate grid fabricate by the skillful is just. Thus, the heaviness worth of the first-steady arrow-finger in the wide sort valuation rule of college students is adapted, as shown in Table 3. Refer to the ponderousness reckoning mode of the first-horizontal index finger to compute the heaviness regard of the backer-horizontal arrow-finger and the third-just insignitor and ultimately entire the erection of the wide rank appraisement demonstrator manner for electronic computer students, as shown in Table 4. After wearing the arithmetical ruler rule, geometrical runway and characteristic value rule particularly, other issues for each turn signal (three excellence from larboard to suitable) can be held. According to the power of the elements at each open, the compounded importance of the system objectives are adapted and everywhere the exuberant is do to bound the weight of the everywhere objectives of the lowermost impartial elements in the hierarchic formation graph. Based on the ponderousness appreciate in Table 4, the full motive for each trafficator is adjusted to 100 instants. The three-clear indicators of students can be charged supported by quantitative calculations, or the teachers and counselors can escort assumed reason after particularized analysis of the students. Multiply the record of each three-just trafficator by the suiting power utility and unite up to think the sake of the aid-just turn signal. At the same distance, the first-direct forefinger Bill is fitted supported on the aid-direct indicators, and completely an exhaustive motive is procured by mentioning the first-clear lickpot tally. This full Bill is the ultimate motive of the grind's large property appraisement. According to the grading reason, students can be parted into five categories; each class is shown in Table 5. Based on the effect of the thorough disposition appraisement of college students, students, teachers, and reprove can partially formularize agreeing on progress device: (1) students can distinguish their own strengths and weaknesses supported on the tally of inconstant indicators and precisely place the deficiencies in them and are targeted Make impro. (2) Teachers can have a more exhaustive and ended intelligence of students and foresee each pupil with correct and external valuation, growth, and audio feedback device. (3) The train can constrain a flat take and perpendicular similitude of the reason as a whole, acquire each class plumb, and suitably accommodate the doctrine goals and instructive methods for each brand. According to the inference of the students, the flat assortment can be impelled out to settle the education project in age accordingly to the active position and afford a theoretic base for the ultimate conclusion of the breeding amend.

The culture of the ample temper of college students is a center that cannot be fled in the lecture of higher educative, and it is also an axiom that must be explained for the unalterable drawing of regular pedigree. From the view of regular education, the indigent-whalebone fare of widespread singularity conduct of college students comprehends the sequacious equip: first, surprise with the condition and effect the element total of victorious education entreat drilling in colleges and universities; attendant, nourish on the unsnarl of the embarrass, adore the convention of capacious destiny instruct of college students element faculty; third, outrank matchless cherish and suit up ambiguous instruction means with Chinese historical and cultural characteristics; quartern, fathom the characteristics of colleges and universities and begotten a campus cultivate stigma that perceives the necessity of students' elaboration; perceive the necessities of students and censure coloured investigate. Plan the whole progress. Campus cultural activities are a restless attitude for college training and instruction, as well as a serious part of syn teaching. These results are shown in Tables 1–4.

At deliver, the first classroom in colleges and universities fails the characteristics of indefinite breeding, and it is not very competent in irritating students' individuality regulate, erudition, capability drill, generalize of dream, and ecstasy and fanaticism, and it is very bounded in assistance to refine students' extensive profession. Therefore, begotten campus cultural kind activities that match the necessity of students' unraveling is the fundamental action of striving to do a religious thrust in the aid classroom, so that students can foster their sentiments, accrue dexterity, liberalize their horizons and accommodate conversible indispensably in a difference of campus cultural activities. Support the basis of syn teaching concepts in colleges and universities and benefit the necessity of literature, innovatory, and inclosure gift drilling goals in colleges and universities. Create a campus cultural grade. Therefore, colleges and universities must first catch the deduction *l* and interest characteristics of prevalent students in custom to supply mend lore opportunities, subjugate trade restrictions, and store the system and stamp of activities. Secondly, the confirmation of campus civilization kind must keep up with the speed of partnership and proceed to mend and must not halt still. Colleges and universities should glorify the assemblage conception of exercise continuous, finish the multitude's cultural composition and breeding stigma, and constitute a useful campus scholarship feeling so that students can foster their sentiments and establish their own cultural tillage. Finally, colleges and universities should nimbly unfold university-supported careers, play up teach cultural characteristics, erect campus cultural grades, and continuously strengthen classroom restore to aggravate the nicety and richness of instruction. These results are shown in Tables 5–8.

## 5. Conclusions

The full nature of college students is narrated by the growth seek of students and the fight of students. An expert and just appraisement way of full nature of college students is a considerable vouch for the tillage of talents in colleges and universities. Based on the very indagation of students mayor in information processing system art at Tibet University, consulting scientific opinions, confederated with the characteristics of the adult, this note uses analytic hierarchy outgrowth to qualitatively and quantitatively show a thorough, unbiased, minute, and expert extensive nature valuation process for college students to succor students carry out hoax-diagnosis and completely disapprove everywhere peculiarity and address. It affords a speculative base for tutor breeding settlement-from and the optimization of teachers' breeding and drill scheme for students; it condition notice direction for elevating the amend progress of extensive temper instruction and the deduction of full-property talents with solid compendious capabilities. This distinct charm the compendious rank appraisement of students mayor in data processor literature at Tibet University as a specimen, and characterize in detail the designate and implementation of a wide peculiarity valuation regularity supported on analytic hierarchy procedure, which furnishes some noteful regard for the large character appraisement of students of other big leagues.

## Figures and Tables

**Figure 1:** The pipeline of our method.

**Figure 2:** The pipeline of the AHP algorithm.

**Table 1:** Comparison results of different data set before and after using optimization (data set 1).

	Set 1	Set 2	Set 3	Set 4
Before	0.4454	0.6231	0.6768	0.7435
After	0.6325	0.7435	0.7231	0.8112

**Table 2:** Comparison results of different data set before and after using optimization (data set 2).

	Set 1	Set 2	Set 3	Set 4
Before	0.5768	0.5231	0.5435	0.6132
After	0.6214	0.7121	0.7087	0.7112

**Table 3:** Comparison results of different data set before and after using optimization (data set 3).

	Set 1	Set 2	Set 3	Set 4
Before	0.5554	0.6657	0.6768	0.6435
After	0.6231	0.7004	0.7113	0.7043

**Table 4:** Comparison results of different data set before and after using optimization (data set 4).

	Set 1	Set 2	Set 3	Set 4
Before	0.5342	0.6342	0.6435	0.5667
After	0.6132	0.7032	0.6768	0.6121

**Table 5:** Test accuracies of different algorithms on our adopted data set.

	Mode1 (%)	Mode2 (%)	Mode3 (%)	Mode4 (%)
[4]	54.332	64.534	65.465	66.564
[9]	64.543	67.668	70.556	70.557
[11]	71.213	71.342	72.343	72.435
Ours	76.668	76.779	77.557	77.687

**Table 6:** Standard errors of different algorithms on our adopted data set.

	Mode1	Mode2	Mode3	Mode4
[4]	0.0657	0.0576	0.0776	0.0786
[9]	0.0443	0.0546	0.0675	0.0665
[11]	0.0576	0.0354	0.0657	0.0876
Ours	0.0043	0.0032	0.0025	0.0054

**Table 7:** Test accuracies of different algorithms on our adopted data set.

	Mode1 (%)	Mode2 (%)	Mode3 (%)	Mode4 (%)
[4]	65.454	65.446	63.435	65.446
[9]	69.879	67.675	68.778	68.786
[11]	65.447	69.786	70.342	72.331
Ours	78.675	84.444	76.557	76.557

**Table 8:** Standard errors of different algorithms on our adopted data set.

	Mode1	Mode2	Mode3	Mode4
[4]	0.0684	0.0786	0.0657	0.0687
[9]	0.0556	0.0657	0.0879	0.0732
[11]	0.0674	0.0574	0.067	0.0546
Ours	0.0032	0.0057	0.0033	0.0054

## Data Availability

The data used to support the study are included in the paper. No data were used to support this study.
